The article "Clinical Study on Long-Term Sinus Reversion Rate and Left Atrial Function Recovery of Mitral Valve Disease with Atrial Fibrillation under Modified Surgical Radiofrequency Ablation" was retracted in 2023. Reasons: signs of a paper mill; suspected computer-generated content; unreliable results or conclusions; concerns about the data.

# Clinical Study on Long-Term Sinus Reversion Rate and Left Atrial Function Recovery of Mitral Valve Disease with Atrial Fibrillation under Modified Surgical Radiofrequency Ablation

**DOI:** 10.1155/2021/5667364

**Published:** 2021-07-06

**Authors:** Jingle Cui, Ziyang Hu, Tao Li, Ziyang Guo, Weiquan Luo, Zhiyong Huang

**Affiliations:** ^1^Department of Cardiothoracic Surgery, Hospital of Traditional Chinese Medicine of Zhongshan, ZhongShan City 528400, China; ^2^Department of Cardiology, Hospital of Traditional Chinese Medicine of Zhongshan, ZhongShan City 528400, China; ^3^Department of Ultrasound, Hospital of Traditional Chinese Medicine of Zhongshan, ZhongShan City 528400, China

## Abstract

We aimed to study the long-term sinus reversion rate and recovery of left atrial function after modified surgical radiofrequency ablation for permanent atrial fibrillation caused by mitral valve disease. From March 2014 to May 2020, 35 patients who underwent modified surgical radiofrequency ablation during cardiac valve surgery in our hospital were selected as the study group, and 25 normal individuals without cardiac structural changes were selected as the control group. The time of modified surgical radiofrequency ablation and long-term sinus reversion rate were measured, and left atrial anteroposterior, superoinferior, left and right diameters, left atrial ejection fraction, left atrial filling index, and left atrial ejection force were measured before and 6 months after surgery. The mean ablation time was 23.2 min, and the long-term sinus reversion rate was 80.0%. The left atrium diameter decreased and the left atrium ejection fraction increased after the operation (*P* < 0.05). The left atrium filling index and ejection force were significantly increased in 28 patients with sinus reversion (*P* < 0.05). The decrease in left atrial diameter and the increase in left atrial ejection fraction were correlated with sinus conversion after surgery (*P* < 0.05). The modified operation is simple, the curative effect is definite, and the sinus reversion rate is high, which is beneficial to the restoration of left atrial structure, ejection function, and hemodynamic function.

## 1. Introduction

Atrial fibrillation is a common arrhythmia that is mostly secondary to valvular heart disease. Due to structural changes in the left atrium after valvular disease, atrial fibrillation often appears persistent. The main treatment for persistent atrial fibrillation is maze III surgery, with a success rate of 97%, but the operation is complex and traumatic [1]. Developments in technology have enabled radiofrequency ablation to be used instead of cutting and suturing. The ablation route is constantly improved and simplified, and the trauma is greatly reduced. The sinus reversion rate can reach 80–90% [2–4]. Studies have shown that atrial fibrillation has a great impact on left atrial function. In addition to structural measurement, mechanical ejection function, hemodynamics, and other indicators have been added to the detection of left atrial function [5–7]. Many studies have investigated the recovery of left atrial function in patients with paroxysmal atrial fibrillation after interventional ablation [8–11], but there are few reports on the recovery of left atrial function after surgical treatment of valvular disease combined with atrial fibrillation [12–14]. In this study, patients with valvular disease complicated by atrial fibrillation were selected as the study subjects. The modified ablation route and procedure was used to treat atrial fibrillation, while surgery was performed on the heart valve. The effect of the modified procedure in shortening the operation time, ensuring a curative effect and the recovery of left atrial function, is discussed.

## 2. Materials and Methods

### 2.1. General Data

From March 2014 to May 2020, 35 patients with mitral valve disease combined with atrial fibrillation underwent mitral valve replacement or plasty and modified maze radiofrequency ablation in our hospital. There were 15 men and 20 women with an average age of 55 years (range, 40–69 years). There were 9 cases of simple mitral valve disease, 18 cases of mitral valve combined with tricuspid valve disease, and 8 cases of mitral valve, aortic valve, and tricuspid valve combined disease. Twenty-five healthy individuals without cardiac structural lesions were selected as the control group. All patients were diagnosed by transthoracic echocardiography before surgery, and left ventricular ejection fraction (LVEF) and left atrial function were measured. The patients were treated with digoxigenin, furosemide, and amiodarone for 1-2 weeks. This study was approved by Zhongshan Hospital of Traditional Chinese Medicine. Written informed consent was obtained from the patient.

### 2.2. Procedure and Radiofrequency Ablation Route

Catheter drainage of the superior vena cava and inferior vena cava was used to establish cardiopulmonary bypass. The right superior and inferior pulmonary vein entrances were ablated under parallel circulation. After cardiac arrest, the left atrium was examined. If a thrombus was present, the thrombus was removed first. The left superior and inferior pulmonary vein entrances were ablated. The left atrial appendage was then excised. The left atrial appendage to the left superior pulmonary vein was ablated, and the left atrial appendage stump was sutured. If a thrombus was found in the left atrial appendage or if the patient was elderly (over 65 years old), ablation was performed at the root of the left atrial appendage and from the right superior pulmonary vein to the root of the left atrial appendage. The left atrial appendage was closed in the left atrium without removal of the left atrial appendage. Next, ablation of the right superior pulmonary vein to the left superior pulmonary vein was performed. The right superior pulmonary vein to the left inferior pulmonary vein was then ablated with ablation forceps around the lateral side of the right inferior pulmonary vein. In the same way, the right superior pulmonary vein to the mitral annulus was ablated. Subsequently, coronary sinus to isthmus ablation was performed. The right atrial incision was sutured as the eighth line. Each ablation line was ablated two to three times (Figure 1). Valve surgery was performed after radiofrequency ablation. An epicardial temporary pacemaker was placed. The ablation equipment used was bipolar radiofrequency ablation forceps (AtriCure Inc.). Ablation energy and time were calculated by an ablation machine according to tissue thickness.

### 2.3. Postoperative Treatment and Follow-Up

The patients were treated with vasoactive drugs to maintain hemodynamic stability and amiodarone to maintain sinus rhythm. An epicardial temporary pacemaker was set to 80 beats per minute to guarantee heart rate. The same drug treatment as before surgery was maintained until 3–6 months after surgery. Six months after the operation, the patients were followed up with electrocardiography and color Doppler ultrasonography. The LVEF, left atrial function including left atrial structure (anterior and posterior, upper and lower, left and right diameters), mechanical function (diastolic and systolic volumes of left atrium were measured by four-chamber echocardiography, and left atrial ejection fraction (LAEF) was calculated), E peak, A peak, and their velocity time integral were measured by color Doppler ultrasound. Left atrial filling index (LAFI) was defined as LAFI = A peak time velocity integral/(A peak time velocity integral + E peak time velocity integral), and left atrial ejection force (AEF) was defined as AEF= 0.5 × *ρ* × MVA × (VA) 2 × 10 − 3, where *ρ* is the viscosity coefficient 1.06/m^3^, MVA is the area of mitral valve orifice (cm^2^) measured using the pressure half-time method, VA is the A peak flow velocity of mitral valve orifice (cm/s), and the unit is kdynes [8]. At the same time, the left atrial function was measured in the 25 controls.

### 2.4. Statistical Methods

SPSS (version 16.0) was used to process the data. Statistical data were expressed as mean ± standard deviation. Statistical significance was set at *P* < 0.05.

## 3. Results and Discussion

### 3.1. Surgery

All patients underwent radiofrequency ablation of atrial fibrillation. In mitral valve replacement, mechanical valve replacement was performed in 18 cases, bioprosthetic valve replacement in 12 cases, and mitral valvuloplasty in 7 cases. The average postoperative discharge time was 19 days. All patients were followed up for 6 months. The mitral valve membrane worked well, without stenosis or regurgitation. During the follow-up period, there were no instances of need to install a permanent pacemaker, stroke, or thrombosis complications. The average ablation time was 23.2 min. Of 35 cases, 28 cases converted to sinus rhythm 6 months after the operation, and the cardioversion rate was 80%.

### 3.2. Left Atrial Structure and Function

The results showed that the left atrial anteroposterior diameter and superoinferior diameter were decreased (*P* < 0.005), and LAEF was increased (*P* < 0.005) (Table 1); there was no significant difference between left and right atrial diameters (*P*=0.139), but the difference was shown in paired analysis (*P*=0.041). There were significant differences in left atrial structure and LAEF before and after the operation in paired analysis (*P* < 0.05).

### 3.3. LAFI and Left AEF

Sinus rhythm was restored in 33 patients after treatment, and A peak was restored. The left atrial filling index and left AEF were calculated from A peak to evaluate left atrial hemodynamics. The LAFI and left AEF increased significantly after sinus reversion, but there was still a significant difference compared with the control group (*P* < 0.05) (Table 2).

### 3.4. Correlation Analysis

There was no significant correlation between the size of the preoperative structure and sinus reversion of atrial fibrillation. There was a correlation between the decrease in the left atrial superoinferior diameter and the increase in LAEF (*P* < 0.05) (Table 3).

## 4. Discussion

In structural heart disease, mitral valve disease often causes atrial fibrillation, which may be caused by an increase in left atrial load and blood stasis resulting from mitral stenosis, and the impact of high-speed systolic blood flow from the left ventricle is caused by mitral regurgitation, both of which eventually lead to the enlargement of the left atrial structure and the formation of multiple reentry pathways in the left atrium. The treatment of atrial fibrillation has changed from the traditional “cut and sew” Cox maze III procedure to current radiofrequency ablation. Among them, bipolar radiofrequency ablation is effective with fewer side effects, and the ablation circuit is constantly improved. The maze radiofrequency ablation in this study followed the Cox maze III procedure; except that, while the right atrial longitudinal incision was “cut and sew” and the ablation route was simplified, the rest of the lines were radiofrequency ablation. Using this improved method, the right lower pulmonary vein incision can be omitted in the operation. Most patients had the left atrial appendage in the heart sutured, which reduced the risk of bleeding. The shortening of operation time plays an important role in myocardial protection and prevention of ischemia-reperfusion injury [15], and microvessels play an important role in myocardial protection [16, 17]. Studies have shown that mitochondrial homeostasis and quality promote myocardial protection [18–20] and reduce myocardial injury [21, 22]. In general, the improved operation method has an improved outcome, simpler operation, shorter operation time, and less frequent bleeding complications than the traditional method.

With the development of atrial fibrillation research, increasing attention has been paid to the role of left atrial function in cardiac function. Atrial fibrillation makes left atrial autonomic systolic function disappear, reducing the length of the left ventricular diastolic period, resulting in a change in cardiac stroke output, which affects the stability of hemodynamics, and leads to a decline in cardiac function. In the past, left atrial function was evaluated using echocardiography only in the structure. In recent years, the study of the left atrial function has changed from simple structure measurement to mechanical ejection function and hemodynamics. In this study, we measured the anterior and posterior diameters of the left atrium in the long axis view of the left heart, superior and inferior diameters, and left and right diameters of the left atrium in the four-chamber view. The LAEF was calculated from the changes in left atrial diastolic and systolic volume in the four-chamber view, the LAFI was calculated from the proportion of A peak area to evaluate the role of left atrial active contraction in the whole left ventricular diastolic period, and the left AEF was calculated from the maximum A peak velocity and mitral orifice area to infer the left atrial active systolic force. The above method is simple and can be used to evaluate left atrial function from multiple perspectives. However, there is no comprehensive index to evaluate left atrial function, and the LAEF is considered to be a more intuitive index.

With respect to left atrial structure and function recovery, paired analysis showed that the left atrial structure and LAEF improved in the long term after the modified ablation. Recovery of the A peak is very important for the evaluation of left atrial hemodynamics. Compared with the patients without cardioversion, the left atrial structure and ejection function of the patients with cardioversion were better, and the left atrial filling index and left AEF were also significantly increased. Some studies have shown that the left atrial function of pure atrial fibrillation can return to normal after interventional radiofrequency ablation [8–11], but that the left atrial function of valvular fibrillation cannot be restored after surgical ablation. The reason is that the left atrial structure of the former has no obvious change, while the left atrial structure of the latter has been enlarged due to the long-term volume overload caused by mitral valve disease. In our study, there was a certain difference from the normal group, indicating that the structural change in the left atrium caused by valvular disease is a chronic remodeling process; although mitral valve disease has been treated and sinus rhythm has been restored, left atrial structure and function are still difficult to return to normal levels. From the correlation analysis, we can see that the more obvious the change in left atrial structure, the lower the possibility of cardioversion. Therefore, the success rate of cardioversion can be predicted by changes in the left atrial structure. In view of the limited number of cases in this study, more cases and further data analysis are needed to support this conclusion.

## 5. Conclusions

In general, modified surgical radiofrequency ablation is simple, the curative effect is definite, and the sinus reversion rate is high, which is beneficial to the restoration of left atrial structure, ejection function, and hemodynamic function. The modified operation is worth clinical promotion.

## Figures and Tables

**Figure 1:** Graphical representation of procedure and radiofrequency ablation route. (a) Superior vena cava. (b) Inferior vena cava. (c) Right atrium. (d) Coronary sinus. (e) Left atrium. (f) Pulmonary venous orifice. (g) Left atrial appendage. (h) Mitral orifice.

**Table 1:** Comparison of left atrial structure and ejection fraction before and 6 months after operation.

	Before operation	6 months after operation	Normal group
Anteroposterior diameter (mm)	51.2 ± 9.2	45.0 ± 8.3 (*P* < 0.005)	36.8 ± 3.4
Superoinferior diameter (mm)	71.7 ± 12.4	59.7 ± 10.0 (*P* < 0.005)	48.0 ± 4.9
Left-right diameter (mm)	53.6 ± 15.0	49.2 ± 8.9 (*P*=0.041)	37.2 ± 3.1
LAEF (%)	19.15 ± 7.9	26.1 ± 8.4 (*P* < 0.005)	55.9 ± 7.2

**Table 2:** Left atrial filling index and left atrial ejection force in the sinus reversion group.

	Postoperative sinus reversion group	Normal group
LAFI (%)	18.6 ± 9.1	36.8 ± 7.5
Left AEF (kdynes)	6.0 ± 4.5	9.7 ± 5.0

**Table 3:** Correlation analysis of postoperative sinus recovery, left atrial structure, and left atrial ejection fraction.

	Anteroposterior diameter	Superoinferior diameter	Left-right diameter	LAEF
Correlation coefficient	−0.158	−0.288^*∗*^	−0.219	0.290^*∗*^
*P*	0.273	0.045	0.131	0.041

Kendall correlation analysis. *P* < 0.05, statistical difference. ^*∗*^Statistical significance.

## Data Availability

The data used to support the findings of this study are available from the corresponding author upon request.

## References

[1] Reston J., Shuhaiber J. (2005). Meta-analysis of clinical outcomes of maze-related surgical procedures for medically refractory atrial fibrillation. *European Journal of Cardio-Thoracic Surgery*.

[2] McClure G. R., Belley-Cote E. P., Jaffer I. H. (2018). Surgical ablation of atrial fibrillation: a systematic review and meta-analysis of randomized controlled trials. *EP Europace*.

[3] Benussi S., Cini R., Gaynor S. L., Alfieri O., Calafiore A. M. (2010). Bipolar radiofrequency maze procedure through a transseptal approach. *The Annals of Thoracic Surgery*.

[4] Khargi K., Keyhan-Falsafi A., Hutten B. A., Ramanna H., Lemke B., Deneke T. (2007). Surgical treatment of atrial fibrillation. *Herzschrittmachertherapie & Elektrophysiologie*.

[5] Hoit B. D. (2018). Assessment of left atrial function by echocardiography: novel insights. *Current Cardiology Reports*.

[6] Ancona R., Comenale Pinto S, Caso P (2014). Left atrium by echocardiography in clinical practice: from conventional methods to new echocardiographic techniques. *The Scientific World Journal*.

[7] Nakagawa M., Saikawa T. (2013). Echocardiogram in atrial fibrillation. *Nihon Rinsho*.

[8] Donal E., Ollivier R., Veillard D. (2010). Left atrial function assessed by trans-thoracic echocardiography in patients treated by ablation for a lone paroxysmal atrial fibrillation. *European Journal of Echocardiography*.

[9] Chin J. Y., Youn H.-J. (2014). The effect of ablation for paroxysmal atrial fibrillation on left atrial volume and function: a one-year follow-up study. *Yonsei Medical Journal*.

[10] Kim J.-S., Im S. I., Shin S. Y. (2017). Changes in left atrial transport function in patients who maintained sinus rhythm after successful radiofrequency catheter ablation for atrial fibrillation: a 1-year follow-up multislice computed tomography study. *Journal of Cardiovascular Electrophysiology*.

[11] Njoku A., Kannabhiran M., Arora R. (2018). Left atrial volume predicts atrial fibrillation recurrence after radiofrequency ablation: a meta-analysis. *EP Europace*.

[12] Chen M.-C., Chang J.-P., Chang H.-W. (2005). Clinical determinants of sinus conversion by radiofrequency maze procedure for persistent atrial fibrillation in patients undergoing concomitant mitral valvular surgery. *The American Journal of Cardiology*.

[13] Wu C.-C., Chang J.-P., Chen M.-C., Cheng C.-I., Chung W.-J. (2017). Long-term results of radiofrequency maze procedure for persistent atrial fibrillation with concomitant mitral surgery. *Journal of Thoracic Disease*.

[14] Chen M.-C., Chang J.-P., Guo G. B.-F., Chang H.-W. (2001). Atrial size reduction as a predictor of the success of radiofrequency maze procedure for chronic atrial fibrillation in patients undergoing concomitant valvular surgery. *Journal of Cardiovascular Electrophysiology*.

[15] Heusch G. (2019). Coronary microvascular obstruction: the new frontier in cardioprotection. *Basic Research in Cardiology*.

[16] Hughes W. E., Beyer A. M., Gutterman D. D. (2020). Vascular autophagy in health and disease. *Basic Research in Cardiology*.

[17] Cuijpers I., Simmonds S. J., van Bilsen M. (2020). Microvascular and lymphatic dysfunction in HFpEF and its associated comorbidities. *Basic Research in Cardiology*.

[18] Wang J., Toan S., Zhou H. (2020). New insights into the role of mitochondria in cardiac microvascular ischemia/reperfusion injury. *Angiogenesis*.

[19] Wang J., Toan S., Zhou H. (2020). Mitochondrial quality control in cardiac microvascular ischemia-reperfusion injury: new insights into the mechanisms and therapeutic potentials. *Pharmacol Res*.

[20] Zhou H., Toan S., Zhu P., Wang J., Ren J., Zhang Y. (2020). DNA-PKcs promotes cardiac ischemia reperfusion injury through mitigating BI-1-governed mitochondrial homeostasis. *Basic Research in Cardiology*.

[21] Sawashita Y., Hirata N., Yoshikawa Y., Terada H., Tokinaga Y., Yamakage M. (2020). Remote ischemic preconditioning reduces myocardial ischemia-reperfusion injury through unacylated ghrelin-induced activation of the JAK/STAT pathway. *Basic Research in Cardiology*.

[22] Tan Y., Mui D., Toan S., Zhu P., Li R., Zhou H. (2020). SERCA overexpression improves mitochondrial quality control and attenuates cardiac microvascular ischemia-reperfusion injury. *Molecular Therapy-Nucleic Acids*.

